# The Evaluation of Clinical Status of Endoscopic Retrograde Cholangiography for the Placement of Metal and Plastic Stents in Cholangiocarcinoma Therapy

**DOI:** 10.1155/2022/5741437

**Published:** 2022-10-11

**Authors:** Min Gong, Qiang Li, You Xu, Yunhui Fu

**Affiliations:** Department of Gastroenterology, Jiangxi Pingxiang People's Hospital, Pingxiang 337055, Jiangxi, China

## Abstract

**Objective:**

Cholangiocarcinoma is a common malignant tumor that occurs in the bile duct system, which can be treated by using the endoscopic retrograde cholangiography (ERCP). This study was aimed at exploring the therapeutic effect of ERCP with metal stent and plastic stent for cholangiocarcinoma.

**Methods:**

The clinical data of 71 patients with cholangiocarcinoma treated by ERCP in our hospital from June 2020 to October 2021 were retrospectively analyzed. According to different stent types, the patients were divided into plastic stent group (*n* = 43) and metal stent group (*n* = 28). Patients in the plastic stent group and metal stent group were received with plastic stent and metal stent, respectively. The indexes of liver function (serum alkaline phosphatase (ALT), direct bilirubin (DBIL), glutamic oxaloacetic transaminase (AST), alkaline phosphatase (ALP), and total bilirubin (TBIL)), postoperative complications, success rate of stent implantation, and survival time of patients in the two groups were determined. Logistic multivariate regression analysis was used to analyze the prognostic factors of postoperative cholangiocarcinoma.

**Results:**

The liver function indexes of the two groups were significantly improved after treatment with the stent, in which the ameliorative effect in the metal stent group was better than that in the plastic stent group (*P* < 0.05). The incidence of postoperative complications in the plastic stent group and the metal stent group was 53.49% and 14.29%, respectively, and the success rate of stent placement was 60.47% and 96.43%, respectively. The incidence of complications in the metal stent group was lower than that in the plastic stent group, and the success rate of stent placement was higher than that in the plastic stent group (*P* < 0.05). The median survival time of patients in the plastic stent group and the metal stent group was 8.15 and 11.83 months, respectively. The survival time of patients in the metal stent group was longer than that of the plastic stent group. The median survival time of patients with types I, II, III, and IV was 12.73, 11.54, 10.57, and 9.36 months, respectively. The survival time of patients with stage I was significantly higher than that of patients with types II, III, and IV. There was an inverse relationship between the disease type and the survival time of patients. Logistic multivariate regression analysis showed that tumor diameter ≥ 5 cm, portal vein invasion, lymph node metastasis, and classification of hilar cholangiocarcinoma were the risk factors (*P* < 0.05) and metal stent type was the protective factor (*P* < 0.05).

**Conclusion:**

In the clinical treatment of patients with cholangiocarcinoma, the placement of metal stent and plastic stent under ERCP plays an important role. The placement of the metal stent under ERCP has a higher success rate and better prognosis and can prolong the survival time of patients to a greater extent, but the price of the metal stent is relatively expensive. For patients with an expected survival period of more than 4-6 months, the metal stent should be considered; otherwise, the plastic stent can be used to maintain cost-effectiveness. Therefore, it is necessary to comprehensively analyze the patient's economic affordability, expected survival time, stent drainage time, and personal needs and then select an appropriate treatment method.

## 1. Introduction

Cholangiocarcinoma is the malignant tumor originating from the extrahepatic bile duct, including the bile duct from the hilar area to the lower segment of the common bile duct. As a common malignant tumor disease, cholangiocarcinoma occurs in the bile duct system with incompletely defined etiology. It is generally believed that the cause of the disease is related to diseases such as bile duct stones and primary cirrhotic cholangitis. In addition, smoking and drinking are the main causes. Cholangiocarcinoma usually occurs in people aged 50-70 years with slight preference in males. Patients have no special clinical symptoms in the early stage of the disease. With the prolongation of the disease time, the patients will have clinical symptoms such as fever, abdominal pain, fatigue, jaundice, and loss of appetite [1]. At present, cholangiocarcinoma is mainly treated by nutritional support, surgery, radiotherapy and chemotherapy, and interventional therapy [2]. Palliative biliary drainage is commonly used in patients with unresectable cholangiocarcinoma to relieve obstructive jaundice, pruritus, or pain to prolong survival. In recent years, with the development of endoscopic technology, endoscopic retrograde cholangiography (ERCP) stent placement has been gradually applied in clinical practice. ERCP stent placement is first used for clinical treatment in 1979. ERCP stent placement has replaced some surgical operations in the treatment of biliary and pancreatic diseases. It is a minimally invasive interventional treatment and has become the main method for the treatment of cholangiocarcinoma [3].

In this study, the placement of metal and plastic stents in ERCP can effectively relieve the symptoms of obstructive jaundice in patients with obvious advantages. In addition, patients with the placement of stents in ERCP display high postoperative survival rate with no obvious damage, lower pain degree than traditional treatment, and safer treatment, which make it being with broad prospect of clinical application. Biliary stents can be divided into metal stents and plastic stents according to the different materials of the implanted biliary stent. Each has its own advantages and disadvantages. When choosing the type of stent placement, the extent and degree of the lesion should be considered, and the patient survival time and stent drainage time should be fully estimated to obtain a higher benefit ratio. The choice of the number of stents to be placed in the biliary tract is still controversial. In this study, metal stents and plastic stents were placed under ERCP to analyze the safety of the two different stents and their impact on patient survival and long-term prognosis. The reports were as follows.

## 2. Materials and Methods

### 2.1. General Information

The clinical data of 71 patients with cholangiocarcinoma treated by ERCP in our hospital from June 2020 to October 2021 were retrospectively analyzed. According to different stent types, the patients were divided into plastic stent group (*n* = 43) and metal stent group (*n* = 28). This study has been approved by the Ethics Committee of our hospital. The following are the inclusion criteria: (1) the patients were diagnosed as cholangiocarcinoma by B-ultrasound, magnetic resonance, or CT; (2) the patients with distant metastasis or late symptoms confirmed by pathology; (3) the patients could be successfully placed with the stent under the guidance of ERCP; and (4) the patients with the complete clinical medical records, and the patients and their families gave informed consent to participate in this study. The following are the exclusion criteria: (1) the patients with severe impairment of liver, kidney, and spleen function; (2) the patients with systemic tumor disease; (3) the patients with mental or cognitive impairment; (4) the patients who do not meet the surgical indications; and (5) the patient with incomplete clinical data or the researcher who withdrawn halfway. There were 43 cases in the control group, 21 women and 22 men, aged 40-92 years, with an average age of 68.34 ± 5.48, while 28 cases in the study group, 13 women and 15 men, aged 40-92 years, with an average age of 68.58 ± 5.26. There was no significant difference in general information between the two groups (*P* > 0.05). The general information of the two groups is shown in Table 1. The process of general data selection is shown in Figure 1.

### 2.2. Methods

Chest X-ray (X-Ray systems, CGR500, France), cardiopulmonary function (K4b~2, COSME, Italy), coagulation function (CX9ALX, Beckman, USA), blood routine (CX9ALX, Beckman), ECG (MAC5500, GE, USA), and liver function (CX9ALX, Beckman) were examined before operation. If the patient was complicated with other diseases, it needed to consult with other departments to accurately evaluate the operation risk. Patients were forbidden to drink six hours before operation. Half an hour before operation, the patient was anesthetized by giving 50 mg pethidine, 10 mg diazepam, and 10 mg anisodamine. The patient was placed in the left prone position, connected to oxygen inhalation, ECG monitoring, and electrode pads. Under endoscope, the hydrophilic guide wire was inserted into the bile duct until the obstruction site, and the obstruction site, scope, and severity were observed. The length and location of the stenosis were determined by injecting nonionic contrast agents such as iodophor. After dilating the stenosis, gradually advance to the appropriate bile duct position through the catheter, and place the bile duct metal stent and plastic stent on the bile duct obstruction site, respectively, ensuring that both ends of the stent need to exceed the obstruction site by about 1 cm. After the operation, the patients were forbidden to drink and eat. ECG monitoring was performed for 12 hours. The vital signs and abdominal conditions of the patients were observed, and the patients were treated with rehydration and liver protection. Antibiotics were given if biliary tract infection occurred. The patients were followed up for two years after the operation to understand the recovery status of the patient's condition.

### 2.3. Outcome Measures

(1) Before treatment and 24 hours after treatment, 3 mL of fasting venous blood was drawn in the morning. Then, the fasting venous blood was centrifuged at 3000 r/min for 10 min to collect the sera. The levels of serum alkaline phosphatase (ALT), direct bilirubin (DBIL), aspartate aminotransferase (AST), alkaline phosphatase (ALP), and total bilirubin (TBIL) were detected using a 7080 automatic biochemical analyzer [4] (CX9ALX, Beckman) in strict accordance with the instructions.

(2) The number of patients with complications such as stent displacement, intraoperative expansion, postoperative pancreatitis, cholangitis, no decrease in total bilirubin, liver abscess, and bleeding was counted 24 hours after treatment, and the total incidence was calculated.

(3) The patients with cholangiocarcinoma were classified by the Bismuth-Corlette classification method. Type I: the tumor was located below the bifurcation of the common hepatic duct with the communication between the left and right hepatic ducts. Type II: the tumor occupied the confluence of the left and right hepatic ducts without no channel between them. Type III: the tumor invaded one hepatic duct. Therein, the patients with the tumor involved the right liver ducts were defined as type IIIa, while those with tumor involved the left hepatic ducts were defined as type IIIb. Type IV: type IV tumors involved bilateral hepatic ducts. The success rate of stent implantation in patients with different types was counted.

(4) The Mann-Whitney *U* test was used to test the stent patency time in the plastic stent group and the metal stent group. The life table method was used to calculate the overall survival rate of patients, and the Kaplan-Meier method was used to represent the survival curve.

(5) The following prognostic factors were analyzed: age, gender (male and female), smoking history, drinking history, family tumor history, tumor diameter (<5 cm and ≥5 cm), tumor differentiation degree (well differentiated, moderately differentiated, and poorly differentiated), portal vein invasion, lymph node metastasis, and hilar cholangiocarcinoma classification (Bismuth-Corlette classification, including type I, type II, type III, and type IV) were collected from all patients.

### 2.4. Statistical Analysis

The test results were analyzed by SPSS 20.0 software. The measurement data were tested by normal distribution. The data conforming to the normal distribution were expressed as ($\overset{¯}{x}\pm s$) and analyzed through independent sample *t* test. The enumeration data were expressed as % and analyzed through Fisher or *χ*^2^ test. The Kaplan-Meier analysis was used to determine the survival time of patients with different types of stents. Log-rank analysis tested the survival curve. Logistic multivariate regression analysis examined the influencing factors for postoperative prognosis of cholangiocarcinoma. *P* < 0.05 indicated the statistical significance.

## 3. Results

### 3.1. Comparison of Liver Function between the Two Groups

There was no significant difference in liver function between the two groups before the treatment (*P* > 0.05). After the treatment, the liver function indexes of the two groups were both significantly improved, among which the ameliorative effect of the liver function indexes in the metal stent group were notably better than that in the plastic stent group (*P* < 0.05), as shown in Table 2.

### 3.2. Comparison of Postoperative Complications between the Two Groups

The incidence of postoperative complications in the plastic stent group and the metal stent group was 53.49% and 14.29%, respectively. The incidence of postoperative complications in the metal stent group was lower than that in the plastic stent group (*P* < 0.05, Table 3).

### 3.3. Comparison of Stent Implantation Success Rate between the Two Groups

The success rates of stent implantation in the plastic stent group and the metal stent group were 60.47% and 96.43%, respectively (Table 4 and Figure 2).

### 3.4. Comparison of Survival Time between the Two Groups

The median survival time of the plastic stent group and the metal stent group was 8.15 and 11.83 months, respectively. The survival time of the metal stent group was longer than that of the plastic stent group (*P* < 0.05, Figure 3).

### 3.5. Univariate Analysis of Prognostic Factors in Patients with Cholangiocarcinoma

A total of 71 patients with cholangiocarcinoma were divided into the poor prognosis group with 33 cases and into the good prognosis group with 38 cases according to the recurrence and metastasis within two years after operation. Univariate analysis showed that there were significant differences between the poor prognosis group and the good prognosis group in the proportion of family tumor history, tumor diameter, degree of tumor differentiation, portal vein infiltration, lymph node metastasis, classification of hilar cholangiocarcinoma, and stent type (*P* < 0.05, Table 5).

### 3.6. Logistic Multivariate Regression Analysis

The factors with statistical significance in Table 5 were taken as independent variables, and the recurrence and metastasis of patients with cholangiocarcinoma two years after operation were taken as dependent variables for logistic multivariate regression analysis. Logistic multiple regression analysis showed that tumor diameter ≥ 5 cm, portal vein infiltration, lymph node metastasis, and classification of hilar cholangiocarcinoma were all risk factors (*P* < 0.05), while metal stent type was protective factor (*P* < 0.05, Table 6).

## 4. Discussion

Patients with cholangiocarcinoma are prone to malignant obstruction of the biliary tract. If not treated in time, it will threaten the patient's life [5]. The anatomical location of cholangiocarcinoma is relatively special, and the location and symptoms of cholangiocarcinoma are dormant [6]. Clinical treatment by placing bile duct stents under ERCP endoscopy can be consistent with human physiological characteristics, reduce the sense of compression on the bile duct, dredge the bile duct, and improve the quality of life of patients after operation [7]. Metal stent and plastic stent are the main materials of biliary stent, and the polyethylene plastic stent is often used at present. The plastic support has the characteristics of convenient replacement, low price, and easy acceptance by patients. However, the replacement cycle of plastic stents is relatively short, and they need to be replaced every 3-6 months, which is prone to bile sludge adhesion and high bacterial infection rate [8, 9]. In this study, metal stents and plastic stents were placed under ERCP to analyze the safety and the effects on survival cycle and long-term prognosis.

In general, metal stents have obvious advantages, such as convenient operation and high histocompatibility. At present, the clinical application of metal stent is more and more extensive, because it is not easy to block and fall off and has good patency [10]. Nevertheless, compared with plastic stents, metal stents are relatively more expensive and less selective in grass-roots hospitals. At the same time, the advantage of metal stents is not obvious for patients with short expected survival cycle, poor drainage effect, and obvious bile duct invasion [11]. Therefore, it is necessary to consider the situation of patients in all aspects when selecting stent materials [12]. This study analyzed the effect of placing bile duct metal and plastic stents under ERCP on liver function and long-term prognosis of patients with cholangiocarcinoma. The results showed that the liver function indexes of the two groups were both significantly improved after treatment, and the improvement of liver function in the metal stent group was greater than that in the plastic stent group. Placement of bile duct metal stent under ERCP can avoid the impact of bile stasis on patients' liver function, improve the blood flow in patients' liver, reduce the level of serum total bilirubin, and enhance liver metabolic function; thus, it is of great significance for relieving bile duct pressure [13]. The results from the present study showed that metal stent was more effective than plastic stent in improving liver function. Endoscopic operation is the retrograde operation. The hydrophilic guide wire can pass through the narrow part more smoothly, which improves the flexibility of the guide wire and avoids the blindness of puncture [14]. The success rates of stent implantation in the plastic stent group and the metal stent group were 60.47% and 96.43%, respectively, in the present study. The results showed that ERCP endoscopic operation could greatly improve the success rate of stent implantation. However, the pancreatic duct will be compressed during stent implantation, which will lead to intestinal fluid reflux [15]. In addition, biliary tract infection complications may occur due to excessive injection of contrast medium during operation. Therefore, the position of stent placement should be controlled within the range of duodenal papilla to ensure the normal function of sphincter and reduce intestinal fluid reflux and the compression on pancreatic duct [16]. In this study, the incidence of postoperative complications in the plastic stent group and the metal stent group was 53.49% and 14.29%, respectively. The results confirmed that ERCP endoscopic metal stent implantation was more feasible and worthy of palliative treatment.

In recent years, new interventional devices and metal stents have been greatly developed and applied. Metal stents can make up for the disadvantages of plastic support, which mainly includes three types, namely, partially covered self-expanding metal support, self-expanding metal support, and fully covered self-expanding metal support [17]. The metal stent material has high finish and large lumen, which is not easy to adhere to bile sludge and bacteria, and will not contact with bacteria in a large area. The outer layer of the metal stent is covered by bile duct mucosal epithelial cells, which reduces the rate of bacterial infection and the probability of bile duct collateral obstruction and is convenient for placement [18]. This study compared the median survival time of patients in two groups, and the median survival time of the plastic stent group and the metal stent group was 8.15 and 11.83 months, respectively. The results showed that there was an inverse relationship between the stage and survival time. With the continuous progress of the disease, the survival time shows a downward trend, so it is necessary to choose an appropriate way for early treatment to improve the quality of life of patients as much as possible. Logistic multiple regression analysis revealed that tumor diameter ≥ 5 cm, portal vein infiltration, lymph node metastasis, and classification of hilar cholangiocarcinoma were all risk factors (*P* < 0.05), while the metal stent type was protective factor (*P* < 0.05), further confirming the clinical application value of metal stents. Plastic stents are inexpensive and easy to maneuver endoscopically; however, plastic stents have a small inner diameter and are often blocked within the stent due to biliary deposits and bacterial infection. Compared with the plastic stents, the metal stents have wider inner diameter and smoother surface. After placing plastic stents and metal stents in 100 patients with bile hilar cholangiocarcinoma, the median patency period of the metal stent group is 5.56 months, which is significantly higher than that of the plastic stent group of 1.86, and the reintervention rate of the metal stents is significantly higher than that of the plastic stents [19]. Metal stents or plastic stents can still be placed in the original stent even if the metal stent is blocked. However, once placed, metal stents cannot be removed and cost more than plastic stents. Therefore, metal stents should be considered for patients with expected survival beyond 4-6 months; otherwise, plastic stents can be used to maintain cost-effectiveness [20]. This study comprehensively analyzed the therapeutic effect of ERCP endoscopic implantation of stents with different materials on cholangiocarcinoma, which has good clinical significance. At the same time, small sample experiments have been done before this study, which could ensure the smooth progress of the study and provide a good foundation for the treatment of patients.

In conclusion, the placement of bile duct metal stent and plastic stent under ERCP plays an important role in the clinical treatment of patients with cholangiocarcinoma. ERCP placement of bile duct metal stent has higher success rate and better prognosis and can prolong the survival time of patients to a greater extent, but the price is relatively expensive. Therefore, it is necessary to comprehensively analyze the patient's economic affordability, expected survival time, stent drainage time, and personal needs and then select an appropriate treatment method. However, this present study still has some limitations. Research time and sample size both affect the research results. In addition, the subjective operation of the operator and the detailed medical history of the patient might induce the result deviation. Therefore, more qualified samples in the following study will be included and the study time and follow-up time will be appropriately extend to avoid the impact of subjective operation on the accuracy of results as much as possible.

## Figures and Tables

**Figure 1:** Process of general data selection.

**Figure 2:** Comparison of stent implantation success rate between the two groups. (a) The plastic stent group. (b) The metal stent group. The success rates of stent implantation in the metal stent group were higher than that in the plastic stent group (*P* < 0.05).

**Figure 3:** Comparison of survival time between the two groups.

**Table 1:** Analysis of general information of two groups.

General information	The plastic stent group (*n* = 43)	The metal stent group (*n* = 28)	*χ* ^2^/*t*	*P*
Gender (female/male)	21/22	13/15	0.039	0.843
Age (year)	68.34 ± 5.48	68.58 ± 5.26	0.183	0.855
Biliary stricture length (cm)	3.24 ± 0.87	3.22 ± 0.92	0.093	0.927
Albumin (<35/≥35 g/L)	15/28	9/19	0.057	0.811
Preoperative GGT (U/mL)	475.32 ± 29.54	476.51 ± 29.63	0.166	0.869
Total bilirubin (ummol/L)			0.470	0.791
≥427	9 (20.93)	6 (21.43)		
342-427	26 (60.47)	15 (53.57)		
205-342	8 (18.60)	7 (25.00)		

**Table 2:** Comparison of liver function between the two groups ($\overset{¯}{x}\pm s$).

Groups		ALT (U/L)	DBIL (*μ*mol/L)	AST (U/L)	ALP (U/L)	TBIL (*μ*mol/L)
The plastic stent group (*n* = 43)	Before treatment	105.24 ± 4.26	165.24 ± 12.85	67.52 ± 6.58	438.52 ± 27.41	164.52 ± 12.73
	After treatment	59.65 ± 3.25^a^	53.24 ± 3.57^a^	34.84 ± 4.28^a^	135.41 ± 11.54^a^	53.42 ± 2.57^a^

The metal stent group (*n* = 28)	Before treatment	105.18 ± 4.23	165.38 ± 12.87	67.54 ± 6.43	438.41 ± 27.44	163.92 ± 12.84
	After treatment	56.42 ± 3.17^ab^	50.37 ± 3.16^ab^	30.21 ± 3.16^ab^	110.39 ± 11.51^ab^	48.46 ± 2.13^ab^

Note: ^a^*P* < 0.05 compared with the same group before treatment. ^b^*P* < 0.05 compared with the plastic stent group after treatment.

**Table 3:** Comparison of postoperative complications between the two groups (cases, %).

Groups	The plastic stent group (*n* = 43)	The metal stent group (*n* = 28)	*χ* ^2^	*P*
Stent displacement	6 (13.95)	1 (3.57)	2.057	0.152
Intraoperative expansion	4 (9.30)	1 (3.57)	0.851	0.356
Postoperative pancreatitis	5 (11.63)	1 (3.57)	1.423	0.233
Cholangitis	3 (13.95)	1 (3.57)	2.057	0.152
No decrease in total bilirubin	2 (0.00)	0 (0.00)	1.340	0.247
Liver abscess	1 (0.00)	0 (0.00)	0.661	0.416
Bleeding	2 (4.65)	0 (0.00)	1.340	0.247
Total complication rate	23 (53.49)	4 (14.29)	11.059	<0.001

**Table 4:** Comparison of stent implantation success rate between the two groups (cases, %).

Type	The plastic stent group (*n* = 43)		The metal stent group (*n* = 28)		*χ* ^2^	*P*
	Cases	Success rate	Cases	Success rate		
Type I	7	6 (85.71)	5	5 (100.00)	0.197	0.657
Type II	15	10 (66.67)	9	9 (100.00)	0.683	0.408
Type III	11	6 (54.55)	8	8 (100.00)	2.289	0.130
Type IV	10	4 (40.00)	6	5 (83.33)	1.121	0.290
Total success rete	43	26 (60.47)	28	27 (96.43)	11.589	<0.001

**Table 5:** Univariate analysis of prognostic factors in patients with cholangiocarcinoma.

Prognostic factors		The poor prognosis group (*n* = 33)	The good prognosis group (*n* = 38)	*χ* ^2^	*P*
Age		65.88 ± 10.16	67.26 ± 8.90		

Gender	Male	19 (57.58)	15 (39.47)	2.319	0.128
	Female	14 (42.42)	23 (60.53)		

Smoking history		8 (24.24)	10 (26.32)	0.040	0.841

Drinking history		6 (18.18)	9 (23.68)	1.592	0.207

Family tumor history		6 (18.18)	1 (2.63)	4.806	0.028

Tumor diameter	<5 cm	13 (39.39)	25 (65.79)	6.180	0.013
	≥5 cm	20 (60.61)	13 (34.21)		

Degree of tumor differentiation	Well differentiated	7 (21.21)	3 (7.89)	6.697	0.035
	Moderately differentiated	8 (24.24)	20 (52.63)		
	Poorly differentiated	18 (54.55)	15 (39.47)		

Portal vein infiltration	Yes	19 (57.58)	12 (31.58)	4.853	0.028
	No	14 (42.42)	26 (68.42)		

Lymph node metastasis	Yes	25 (75.76)	15 (39.47)	9.453	0.002
	No	8 (24.24)	23 (60.53)		

Classification of hilar cholangiocarcinoma	Type I	5 (15.15)	14 (36.84)	10.702	0.013
	Type II	9 (27.27)	16 (42.11)		
	Type III	12 (36.36)	6 (15.79)		
	Type IV	7 (21.21)	2 (5.26)		

Stent type	Metal stent	7 (21.21)	21 (55.26)	8.574	0.003
	Plastic stent	26 (78.79)	17 (44.74)		

**Table 6:** Logistic multivariate regression analysis.

Factors	*B*	SE	Wald	*P*	OR	95% CI
Tumor diameter ≥ 5 cm	0.871	0.290	9.105	0.003	2.382	1.352~4.129
Portal vein infiltration	1.496	0.302	24.355	0.0001	4.460	2.452~8.075
Lymph node metastasis	1.110	0.356	10.213	0.001	3.026	1.526~5.972
Classification of hilar cholangiocarcinoma	1.050	0.370	8.084	0.004	2.850	1.372~5.852
Metal stent type	-1.861	0.692	7.238	0.007	0.155	0.040~0.603

## Data Availability

All data, models, and code generated or used during the study appear in the submitted article.
